The article "Human Resource Demand Prediction and Configuration Model Based on Grey Wolf Optimization and Recurrent Neural Network" was retracted in 2023. Reasons: suspected computer-generated content; unreliable results or conclusions; concerns about the data; concerns about the results or conclusions.

# Human Resource Demand Prediction and Configuration Model Based on Grey Wolf Optimization and Recurrent Neural Network

**DOI:** 10.1155/2022/5613407

**Published:** 2022-08-27

**Authors:** Navaneetha Krishnan Rajagopal, Mankeshva Saini, Rosario Huerta-Soto, Rosa Vílchez-Vásquez, J. N. V. R. Swarup Kumar, Shashi Kant Gupta, Sasikumar Perumal

**Affiliations:** ^1^Business Studies, University of Technology and Applied Sciences, Salalah, Oman; ^2^Department of Management Studies, Government Engineering College Jhalawar, Jhalrapatan, Rajasthan, India; ^3^Graduate School, Universidad Cesar Vallejo, Lima, Peru; ^4^Faculty of Science, Universidad Nacional Santiago Antunez de Mayolo, Huaraz, Peru; ^5^MIEEE, Department of Computer Science and Engineering, SR Gudlavalleru Engineering College, Gudlavalleru, India; ^6^Computer Science Engineering, Integral University, Lucknow, UP, India; ^7^Department of Computer Science, Wollo University, Kombolcha Institute of Technology, Kombolcha, Ethiopia Post Box No. 208

## Abstract

Business development is dependent on a well-structured human resources (HR) system that maximizes the efficiency of an organization's human resources input and output. It is tough to provide adequate instructions for HR's unique task. In a time when the domestic labor market is still maturing, it is difficult for companies to make successful adjustments in HR structures to meet fluctuations in demand for human resources caused by shifting corporate strategies, operations, and size. Data on corporate human resources are often insufficient or inaccurate, which creates substantial nonlinearity and uncertainty when attempting to predict staffing needs, since human resource demand is influenced by numerous variables. The aim of this research is to predict the human resource demand using novel methods. Recurrent neural networks (RNNs) and grey wolf optimization (GWO) are used in this study to develop a new quantitative forecasting method for HR demand prediction. Initially, we collect the dataset and preprocess using normalization. The features are extracted using principal component analysis (PCA) and the proposed RNN with GWO effectively predicts the needs of HR. Moreover, organizations may be able to estimate personnel demand based on current circumstances, making forecasting more relevant and adaptive and enabling enterprises to accomplish their objectives via efficient human resource planning.

## 1. Introduction

Demand prediction for human resources (HR) is the practice of estimating the number and quality of personnel that will be required. For the forecast to be an accurate predictor, the annual budget and long-term company plan must be translated into activity levels for each function and department. Human resource demand forecasting is required to appropriately plan HR supply and demand. Implementing an enterprise development strategy may be aided by the development of an accurate human resource demand forecasting model that is linked to the company's growth [1]. When it comes to predicting the needs of an organization's workforce, there are two components: demand and supply. The prediction of demand for HR is a precondition for the forecast of supply of HR. Human resource planning can only be done effectively if the demands of the company's future development are clearly defined because of the company's current situation and the supply and demand of HR. There will be a skill scarcity in the company if there are too many staff demand estimates, and this might impede the company's future growth as well [2]. The purpose of industrial development is to utilize natural resources and energy, as well as human resources, to aid industrial expansion by providing jobs and increasing exports. In today's competitive business world, organizations must continuously think about and adapt to the ever-changing environment to succeed. The company's products must be of the highest possible quality and inventive to meet the demands of a changing market. Competitiveness and long-term sustainability of an organization can only be achieved via the use of total quality management (TQM) and strategic human resource management (SHRM) [3].  Figure 1 depicts human resource planning.

The article "Human Resource Demand Prediction and Configuration Model Based on Grey Wolf Optimization and Recurrent Neural Network" was retracted in 2023. Reasons: suspected computer-generated content; unreliable results or conclusions; concerns about the data; concerns about the results or conclusions.

Figure 1 explains that, to set out a strategy for human resource management, HR experts need a thorough awareness of their firm, as well as the ability to take into account different elements. Seven essential elements in the planning process may be used depending on the specifics of an enterprise: Determining the organization's goals is the first step, compiling a list of current employees is the second step, and the third step is to predict your human resources (HR) requirement; counting the number of skills gaps and their magnitude is the fourth step, making a plan of action is the fifth step, putting the strategy into action and integrating it with other aspects of your life is the sixth step, and monitoring, measuring, and providing feedback represent the final step.

Analyzing objectives is the initial step, inventory current human resources, forecast demand, estimate gaps, formulate plans, implement plans, monitor, control, and give feedback. Accurate forecasts of demand for HR may assist contemporary businesses to identify vacant or overstaffed positions and guide the logical distribution of HR. Because of this, it is important for the long-term viability of companies. It has resulted in various HR information systems developing decision-support functions and exploring ways to use existing HR data to enhance the allocation relationship between the internal staff and post requirements to solve a problem with HR allocation and provide scientific and rational support for the optimal positions [4]. A contemporary company's existence and resource development are dependent on its HR and its most valuable asset. To use HR effectively as well as the value and efficiency of HR is a key indicator of whether an enterprise's HR management has been successful or unsuccessful. Employee career development is becoming a more important aspect of HR growth in the workplace [5].

The article "Human Resource Demand Prediction and Configuration Model Based on Grey Wolf Optimization and Recurrent Neural Network" was retracted in 2023. Reasons: suspected computer-generated content; unreliable results or conclusions; concerns about the data; concerns about the results or conclusions.

The remainder of the article is organized as follows: Section 2 provides a literature review and a problem statement. Proposed techniques are shown in Section 3.  Section 4 contains the results. Section 5 is the discussion.  Section 6 is the proposed work's conclusion.

## 2. Literature Review

According to study of [6], the notion of total quality (TQ) has gained a lot of traction in North America. Line management has always been concerned with total quality, which is based on the concept that firms may prosper by serving the demands of their consumers. Human and industrial relations experts, on the other hand, have been advocating some of the ideas advanced by total quality converters for quite some time. In this context, their involvement in the implementation of a comprehensive quality strategy can only be beneficial. According to study of [7], TQM implementation was shown to be most influenced by “training and education,” “incentive compensation,” and “employee development” policies, according to research that examined the relationship between various HRM practices and TQM adoption. Human resource management adoption has the greatest influence on TQM procedures such as satisfaction of customers, statistical quality assurance, and cultural change and innovation. Also investigated were human resources management and total quality management as part of the research. In organizations that implemented HRM and TQM, “customer satisfaction” and “staff happiness” were strongly linked. According to study of [8], the HR scheduling model is based on the evaluation of HR data and the determination of the job matching score. Afterward, based on the job matching score, workers are scheduled. Grouping operations of neural networks are used as outputs in this study to increase neural network performance. An upgraded neural network is created once the data features are sorted and processed. To get the best possible results, for network configuration, we use a hierarchical paradigm. According to study of [9], HR are an organization's most important asset, and accurate demand forecasting is essential to making the most use of them. Predictive models are used to examine the company's human resource demands and define essential components of human resource allocation, starting with fundamental ideas of forecasting HR. This uses back-propagation neural networks (BPNN) and radial basis function neural networks (RBFNN). Two types of neural networks are used to anticipate current human resource needs based on past data. The outcomes of the predictions may be used by the company's managers to plan and allocate HR in a way that maximizes productivity. According to study of [10], the development of a country is heavily influenced by its HR. To improve the adaptability of specific-level strategy, forecasting demand for HR is done in both the commercial and governmental sectors. In addition, regular employment strengthens macroeconomic stability and fosters a sense of urgency for long-term prosperity. As outlined in this work, we use machine learning to predict the demand for human resources. According to study of [11], both a neural network-based dynamic learning prediction algorithm and an algorithm for optimizing resource allocation are proposed in this article; HR may be organized around just two shifts thanks to these two algorithms, which lessen the unpredictability of ship arrivals. The opposite is also true: operators can be optimally distributed throughout the day, taking into consideration real demand and the terminal's operations. In addition, because these algorithms are based on universal variables, they may be used at any transshipment port. According to study of [12], HR for health planning should be in sync with health scheme requirements for an efficient health system. To support HRH programs and policies, it is necessary to create strategies for quantifying the requirements and supply of health workers. Secondary data on service use and population projections, as well as expert opinions, were the primary sources of information for this investigation. Using the health demand technique, the HRH requirements were estimated based on the anticipated service utilizations. The staffing standard and productivity were used to transform into HRH requirements. According to study of [13], multiskilled HR in R&D projects may be allocated using an optimization model that considers each worker's unique knowledge, experience, and ability. In this approach, three key characteristics of HR are taken into consideration: the various skill levels, the learning process, and the social interactions that occur within working groups. There are two approaches to resolving the multiobjective problem: The optimal Pareto frontier is first explored to find a collection of nondominated solutions, and then, armed with new knowledge, the ELECTRE III approach is used to find the best compromise between the various goals. Each solution's uncertainty is represented by fuzzy numbers, which are then used to calculate the ELECTRE III's threshold values. The weights of the objectives are then calculated based on the relative importance of each objective to the others. According to study of [14], a multiagent approach for allocating HR in software projects that are distributed across many time zones is introduced by work. When a project needs HR, this mechanism takes into account the context of the project participants, the requirements of the activities, and the interpersonal interaction between those people. Contextual information provided by the participants includes things like culture, language, proximity in time, prior knowledge, intelligence collection, and reasoning, and allocation of HR falls within the purview of this system. According to study of [15], the design and implementation of flexible information systems rely heavily on knowledge of how businesses work. There are a variety of procedures that companies go through daily. To carry them out, a series of interconnected events and actions or tasks must be completed. Additionally, it incorporates key decision points and the individuals involved in carrying out the process to provide a final deliverable that comprises one or more outputs. According to study of [16], allocating resources at design time and runtime is a common task for business process management systems to undertake. This study aims to fill up the knowledge gap. User preference models for semantic web services have been proven and versatile; therefore we provide a method to define resource preferences. In addition, we show the approach's practicality by implementing one. According to study of [17], an organization's operations are orchestrated with the help of business process management systems. These systems use information about resources and activities to determine how to distribute resources to accomplish a given task. It is commonly accepted that resource allocation may be improved by taking into account the characteristics of the resources that are being considered. The Fleishman taxonomy may be used to identify activities and HR. To allocate resources throughout the process runtime, these specs are employed. We demonstrate how a business process management system may implement the ability-based allocation of resources and assess the technique in a realistic situation. According to study of [18], one of the most important aspects of an organization's viewpoint is allocating the most appropriate resource to carry out the operations of a business process. The business processes may benefit from increased efficiency and effectiveness if the resources responsible for carrying out the activities are better selected. On behalf of enterprises, we have defined and categorized the most important criteria for resource allocation methodologies. Criteria about HR were the primary focus of our investigation. It is our aim that the proposed classification would aid those in charge of process-oriented systems in discovering the sort of information needed to assess assets. As a result of this categorization, additional resource-related information may be captured and integrated into BPMS systems, which might improve the present support for the organizational viewpoint. Additional criteria for evaluation will be added, and we intend to investigate the effects of those factors on resource allocation and codify the criteria for resource allocation identified in taxonomy of resource allocation criteria. According to studies of [19, 20], human resource allocation is further complicated by the presence of team fault lines, which are detailed in this work. Using the information value, we first examine resource characteristics from a demographic and business process viewpoint before selecting essential qualities and assigning a weight to them. This is followed by qualitative and quantitative analysis of team fault lines based on the clustering results of HR. The base and ensemble performance prediction model is built using a multilayer perception. Subsequently, the allocation model and flow are developed. In a real-world scenario, the rationality and efficacy of our human resource allocation approach employing team fault lines were examined, with findings showing that our method can effectively distribute HR and optimize business processes. According to study of [21], an on-the-fly allocation of HR using Naive Bayes is proposed in this paper. Resource allocation plans are said to be updated and performed “on the fly” in this context, meaning that current human resource performance is taken into account while they are being implemented. Our research shows that the suggested methodology takes less time overall to complete than existing methods of allocating resources. The researchers hypothesized, using a numerous constituency perspective of the HR function, that organizational financial investment in their HR functions will have an impact on labor productivity and that this relationship will be moderated by the presence of professional HR staff and the adoption of high performance work systems [22, 23]. Selection, training, working conditions, and assessment were included as independent variables in this study's analysis of HR planning while job satisfaction as a proxy for organizational performance was used as the dependent variable. A self-rated questionnaire has been issued to the organization's top level, medium level, and lower level managers who have read current and prior extensive literature on the importance of human resource practice in organizations [24].

The article "Human Resource Demand Prediction and Configuration Model Based on Grey Wolf Optimization and Recurrent Neural Network" was retracted in 2023. Reasons: suspected computer-generated content; unreliable results or conclusions; concerns about the data; concerns about the results or conclusions.

### 2.1. Problem Statement

Nonlinearity and unpredictability in each component's relationship to the demand for HR are considerable, as are the incompleteness and inaccuracy of corporate human resource data. However, the workforce planning process reveals that many organizations are unsatisfied with their ability to convert company strategy into the particular numbers of personnel needed to fulfill business objectives. It was commonly thought that demand forecasting, or figuring out how many employees are needed, was one of the most difficult aspects of managing labor shortages. Disaster relief organizations have several challenges, including limited human and financial resources and unpredictability in disaster assistance environments. Despite this, no single demand forecasting model has been established to address the aforementioned issue.

## 3. Proposed Methodology

In this phase, we examine the human resource demand prediction and configuration model based on grey wolf optimization and recurrent neural network.  Figure 2 depicts the overall methodology used.

In Figure 2, the data is collected, and the data can be preprocessed using normalization. Principal component analysis (PCA) is used for feature extraction. A recurrent neural network is used for prediction and grey wolf optimization is used for human resource demand prediction.

### 3.1. Data Collection

The 9,855 unique employee users in our dataset represent nearly 15% of the workforce. Over a year and a half, we gathered all 15,200 communications with clear reply links. We have cleaned up the message content by using a stemming step; after normalization phase, we were able to extract 4,384 unique terms from the text of all communications. Additionally, we have collected information on the companies in which the employees who have signed up for our corporate micro blogging platform have been employed (a subset of the total business hierarchy). We create a profile for each person that provides data on their present and prior roles within the organization, as well as a timeline of their previous work history, projects they worked on, and so on [25].

The article "Human Resource Demand Prediction and Configuration Model Based on Grey Wolf Optimization and Recurrent Neural Network" was retracted in 2023. Reasons: suspected computer-generated content; unreliable results or conclusions; concerns about the data; concerns about the results or conclusions.

### 3.2. Data Preprocessing Using Normalization

Typically, healthcare databases are made up of a range of heterogeneous data sources, and the data extracted from them are different, partial, and redundant, all of which have a significant impact on the final mining outcome. As a result, healthcare data must be preprocessed to guarantee that they are accurate, full, and consistent and have privacy protection. Normalization is a preprocessing approach in which the data are scaled or altered to ensure that each feature contributes equally to the total. It is possible to construct a new range from an existing one using the normalization procedure. Predictions or forecasts based on this information may be very valuable. Each feature contributes the same amount of data whether the raw data are rescaled or transformed. Outliers and dominant features, two significant data problems that impede machine learning algorithms, are addressed here. Based on statistical measurements from raw (unnormalized) data, several ways for normalizing data within a specified range have been devised. We normalized our data using the Min-Max and *Z*-score methods. According to the way raw data statistical characteristics are used to normalize the data, these techniques are categorized.

Min-Max normalization is a technique for converting data linearly at the start of the range. Using this method, the relationship between different pieces of information is preserved. Predefined borders with predefined boundaries are a crucial strategy that can correctly fit information.

Following this approach to normalization,

(1) $$\begin{array}{c} O^{,}=\left(\frac{O-\text{min value of }O}{\text{max value of}O-\text{min value of }O}\right)*\left(R-I\right)+I. \end{array}$$

Min-Max data is included in *O*, and one of the boundaries is [*I*, *R*].

The range of the real data is denoted by *O*, while the mapped data is denoted by *O*.

In the *Z*-score normalization procedure, the mean and SD of the data are used to obtain a normalized value from unstructured information. As can be seen in (2), the unstructured data may be normalized using the *Z*-score variable.

(2) $$\begin{array}{c} f_{l}^{\prime }=\frac{f_{l}-\bar{Z}}{\text{std}\left(Z\right)}, \end{array}$$

where *f*_*l*_′ shows the standardised *Z*-score values and *f*_*l*_ shows which *l*^th^ column's row *Y* the value is in.

(3) $$\begin{array}{c} \text{std}\left(Z\right)=\sqrt{\frac{1}{\left(M-1\right)}\sum_{l=1}^{m}{\left(f_{l}-\bar{Z}\right)}^{2}},\\ \bar{Z}=\frac{1}{m}\sum_{l=1}^{m}f_{l}\text{or mean value.} \end{array}$$

In this example, the variables or columns that begin with “*l*” are found in each of the rows *D*, *E*, *F*, and *G* through *H*. *Z*-score approach may be used in each row since every value in a row is equal, resulting in zero standard deviation, and every value in that row is set at 0 to generate standard data. Min-Max normalization is similar in that it shows the range of values between 0 and 1, as is the Z-score.

The article "Human Resource Demand Prediction and Configuration Model Based on Grey Wolf Optimization and Recurrent Neural Network" was retracted in 2023. Reasons: suspected computer-generated content; unreliable results or conclusions; concerns about the data; concerns about the results or conclusions.

Scaling by decimal points is the method that allows for the range of −1 to 1. In line with this strategy,

(4) $$\begin{array}{c} f^{l}=\frac{g}{10^{s}}. \end{array}$$

Here, *f*^*l*^ indicates the values scaled, *g* represents the value range, and *s* denotes the smallest integer Max(|*f*^*l*^|) < 1.

### 3.3. Feature Extraction Using Principal Component Analysis (PCA)

In this study, we extract features using principal component analysis (PCA), which yields encouraging results.

#### 3.3.1. Principal Component Analysis (PCA)

PCA is a technique for reducing the number of dimensions in a dataset. When a high-dimensional dataset is reduced to a smaller dimension, PCA transforms it into a least-squares projection. Datasets can be reduced in dimensionality by discovering a new collection of variables smaller than the original set that represents the significant primary variability in the data. Most of the sample's information remains intact as PCA extracts essential details from complex datasets. It is a straightforward, nonparametric approach to reducing dimensions. As a result, data compression and categorization can benefit from it. In a wide range of industries, principal component analysis has been utilized. Pattern recognition and other data reduction techniques are good examples of picture processing and compression. Computer-Aided Discrepancy Analysis is a technique for finding the direction of the highest variation within a given input space and calculating the covariance matrix's principal component.

The following is the algebraic definition of PCA.

Calculate the covariance of *Y* and the mean of *Y* for data matrix *Y*.

(5) $$\begin{array}{c} \mu ≔F\left\{Z\right\}, \end{array}$$

Then compute the correlation coefficient.

(6) $$\begin{array}{c} S=\text{COV}\left(Y\right)=F\left\{\left(Y-\mu \right)\right\}\left(\mu \right){\left(Y-\mu \right)}^{N}. \end{array}$$

In order to count the eigenvectors *f*_1_, *f*_2_,…, *f*_*O*_, *j* = 1,2,…, *O* and eigenvalues *λ*_*j*_ of the covariance *S* eigenvalues, sort the values in decreasing order.

Solving the equation for *S*, the covariance

(7) $$\begin{array}{c} \left|\lambda J-S\right|=0. \end{array}$$

Get the eigenvalues by decomposing using SVD.

(8) $$\begin{array}{c} \lambda_{1}\geq \lambda_{2}\geq \wedge ,\geq \lambda_{q}\geq 0. \end{array}$$

With the corresponding eigenvectors, *f*_*j*_ (*j*=1,2, ∧, *q*).

The article "Human Resource Demand Prediction and Configuration Model Based on Grey Wolf Optimization and Recurrent Neural Network" was retracted in 2023. Reasons: suspected computer-generated content; unreliable results or conclusions; concerns about the data; concerns about the results or conclusions.

Counting the first *N* eigenvalues is used to pick *λ*_*j*_ to retrieve the principal components.

(9) $$\begin{array}{c} \frac{\sum_{j=1}^{N}\lambda_{j}}{\sum_{k=1}^{O}\lambda_{j}}. \end{array}$$

The first *N* eigenvalue that increased the cumulative percentage by 85 percent is selected as the major component.

The data are projected into a smaller subspace with fewer dimensions.

(10) $$\begin{array}{c} Q=X^{U}Y. \end{array}$$

We may minimize the number of variables or dimensions from *o* to *N* (*N* ≪ *o*) by utilizing the first *N* respective eigenvectors.

The principal component analysis aims to identify linear combinations of factors that best describe the data. We are experimenting with PCA as a tool for extracting features and shrinking dimensions. We may now experiment with a wide range of various classification or grouping methods based on the data we have acquired.

#### 3.3.2. Recurrent Neural Network (RNN)

We look at probability distributions defined over discrete sample space, with a single configuration consisting of *α* ≡ (*α*_1_, *α*_2_,…, *α*_*O*_) list of *O* variables *α*_*o*_ and *α*_*o*_ ∈ {0,…, *e*_*w*_ − 1}. The input dimension *e*_*w*_ denotes the number of potential values for each variable *α*_*o*_.  Figure 3 shows that.

In circumstances when variables *α*_*o*_ have high correlations, one of the most important tasks in machine learning is to infer probability distributions from a collection of empirical data. We utilize the product rule for probabilities to describe the likelihood of a configuration *α* as *Q*(*α*) ≡ *Q*(*α*_1_, *α*_2_,…, *α*_*O*_).

(11) $$\begin{array}{c} Q\left(\alpha \right)=Q\left(\alpha_{1}\right)Q\left(\alpha_{2}|\alpha_{1}\right)\ldots Q\left(\alpha_{O}|\alpha_{O-1},\ldots ,\alpha_{2},\alpha_{1}\right), \end{array}$$

where *Q*(*α*_*j*_*|α*_*j*−1_,…, *α*_2_, *α*_1_) ≡ *Q*(*α*_*j*_*|α*_<*j*_) is the conditional distribution of *α*_*j*_ given a configuration of all *α*_*j*_ with *k* < *j*.

RNNs are a kind of correlated probability distribution of the form (11), in which *Q*(*α*) is defined by the conditionals *Q*(*α*_*j*_*|α*_<*j*_). A recurrent cell, which has appeared in many forms in the past, is the basic building unit of an RNN.

A recurrent cell is a nonlinear function that transfers the direct sum (or concatenation) of an incoming hidden vector *i*_*o*−1_ of dimension *d*_*i*_ and an input vector *α*_*O*−1_ to output is hidden vector *i*_*o*_ of dimension *d*_*i*_ in the simplest form possible.

(12) $$\begin{array}{c} i_{o}=g\left(X\left[i_{o-1};\alpha_{o-1}\right]+c\right). \end{array}$$

A nonlinear activation function is *g*.

The article "Human Resource Demand Prediction and Configuration Model Based on Grey Wolf Optimization and Recurrent Neural Network" was retracted in 2023. Reasons: suspected computer-generated content; unreliable results or conclusions; concerns about the data; concerns about the results or conclusions.

The weight matrix *X* ∈ *ℝ*^*e*_*i*_×(*e*_*i*_+*e*_*v*_)^, the bias vector *c* ∈ ℝ^*e*_*i*_^, and the states *i*_0_*α*_0_ that initiate the recursion are the parameters of this basic RNN (“vanilla” RNN). We set *i*_0_ and *α*_0_ to constant values in this study. Vector *α*_*n*_ encodes the input *α*_*n*_ in a single pass. The whole probability *Q*(*α*) is computed by successively calculating the conditionals, beginning with (*α*_1_), as follows:

(13) $$\begin{array}{c} p\left(\alpha_{o}|\alpha_{o-1},\ldots ,\alpha_{1}\right)=z_{o}.\alpha_{o}, \end{array}$$

where the right-hand side has the standard scalar product of vectors and

(14) $$\begin{array}{c} {\text{z}}_{o}\equiv T\left(Vi_{o}+d\right). \end{array}$$

*V* ∈ ℝ^*e*_*w*_×*e*_*i*_^ and *d* ∈ ℝ^*e*_*w*_^ are the weights and biases of a Softmax layer, respectively, while *T* is the Softmax activation function.

(15) $$\begin{array}{c} T\left({\text{w}}_{o}\right)=\frac{\text{exp}\left({\text{w}}_{o}\right)}{\sum_{j}\text{exp}\left({\text{w}}_{j}\right)}, \end{array}$$

In (13) *z*_*o*_=(*z*_*o*_^1^,…, *z*_*no*_^*e*_*w*_^) is an *e*_*w*_-component vector of positive, real values that add up to 1.

(16) $$\begin{array}{c} {\text{z}}_{o1}=1. \end{array}$$

Thus, a probability distribution over states *α*_*o*_ is formed. The entire probability *Q*(*α*) is given by

(17) $$\begin{array}{c} Q\left(\alpha \right)=\prod_{n=1}^{O}z_{o}.\alpha_{o}. \end{array}$$

Note that *Q*(*α*) is already properly normalized to unity such that

(18) $$\begin{array}{c} Q{\left(\alpha \right)}_{1}=1. \end{array}$$

The hidden vector *i*_*o*_ encodes information about prior spin configurations *α*_<*o*_, as shown in (12) and (13). History *α*_<*o*_*ɛ* is important for predicting the probability of subsequent *α*_*o*_ for correlated probabilities. The RNN is capable of simulating tightly linked distributions by transmitting hidden states in (13) between sites. The dimension of the concealed state will be referred to as the number of memory units *i*_*o*_.  Figure 3 shows the framework of RNN.

### 3.4. Grey Wolf Optimization (GWO)

The grey wolf optimization (GWO) algorithm is a new bio-inspired optimization approach. The main goal of the GWO method is to find the best solution for a given issue utilizing a population of search agents. The social dominance hierarchy that creates the candidate solution in each iteration of optimization distinguishes the GWO algorithm from other optimization algorithms. Tracking, surrounding, and assaulting the target are the three processes in the hunting mechanism. Thus, GWO stands for the grey wolf's mathematical hunting approach, which is utilized to tackle complex optimization problems. As a result, the best solution to a problem has been deemed a victim.

The article "Human Resource Demand Prediction and Configuration Model Based on Grey Wolf Optimization and Recurrent Neural Network" was retracted in 2023. Reasons: suspected computer-generated content; unreliable results or conclusions; concerns about the data; concerns about the results or conclusions.

The three upper levels' movement represents the victim being encircled by grey wolves, as stated by the following formula:

(19) $$\begin{array}{c} \overset{⟶}{E}=\overset{⟶}{D}.\overset{⟶}{Y_{q}\left(u\right)}-\overset{⟶}{Y}\left(u\right). \end{array}$$

*Y*_*q*_indicates the prey position vector, *Y* represents the grey wolf location, and *D* is the coefficient vector. Using the following equation, the result of vector *E* is used to shift a specific element closer to or away from the region where the optimal solution, which symbolizes the prey, is placed.

(20) $$\begin{array}{c} \overset{⟶}{y\left(t+1\right)}=\left|\overset{⟶}{y_{r}\left(t\right)-\overset{⟶}{c}.\overset{⟶}{d}}\right|,\text{with }\overset{⟶}{c}=2\overset{⟶}{c.}\overset{⟶}{m_{1}-\overset{⟶}{c}}, \end{array}$$

where *s*_1_ is chosen at random from the range [0, 1], and over a predetermined number of repetitions, an is decreased from 2 to 0 . If |B| is greater than one, this corresponds to exploitation behavior and replicates prey attack behavior. If |*B*| > 1, the wolf spacing from the victim is imitated. [−2, 2] are the recommended values for *A*. Using the following mathematical equations, three higher levels, *a*, *b*, and *c*, will be calculated.

(21) $$\begin{array}{c} \overset{⟶}{E_{a}}=\left|\overset{⟶}{D_{1}}.\overset{⟶}{Y_{a}}-\overset{⟶}{Y}\right|\text{with}\overset{⟶}{Y_{1}}=\overset{⟶}{Y_{a}}-\overset{⟶}{Y_{a}}.\left({\overset{⟶}{E}}_{a}\right),\\ \overset{⟶}{E_{b}}=\left|\overset{⟶}{D_{2}}.\overset{⟶}{Y_{b}}-\overset{⟶}{Y}\right|\text{with}\overset{⟶}{Y_{2}}=\overset{⟶}{Y_{b}}-\overset{⟶}{Y_{b}}.\left(\overset{⟶}{E_{b}}\right),\\ \overset{⟶}{E_{c}}=\left|\overset{⟶}{D_{3}}.\overset{⟶}{Y_{c}}-\overset{⟶}{Y}\right|\text{with}\overset{⟶}{Y_{3}}=\overset{⟶}{Y_{c}}-\overset{⟶}{Y_{c}}.\left(\overset{⟶}{E_{c}}\right). \end{array}$$

Assume that *a*, *b*, and *c* have enough information about the likely whereabouts of the victim to mathematically imitate the grey wolf's hunting method. Furthermore, the top three best solutions are preserved, forcing the other agents to update their positions following the best agents *a*, *b*, and *c*. The pseudocode of the GWO is given in Algorithm 1, and this behavior is mathematically represented by the following statement.

(22) $$\begin{array}{c} \overset{⟶}{Y}\left(u+1\right)=\frac{\overset{⟶}{y_{1}}+\overset{⟶}{y_{2}}+\overset{⟶}{y_{3}}}{3}. \end{array}$$

## 4. Result

In this phase, we examine the human resource demand prediction and configuration model based on grey wolf optimization and recurrent neural network. The parameters are in-demand analytics skills, human resource satisfaction index (HRSI), prediction rate, and error rate. The existing methods are convolution neural network (CNN [26]), double cycle neural network (DCNN [27]), whale optimization (WO [8]), and particle swarm optimization (PSO [28]).

The article "Human Resource Demand Prediction and Configuration Model Based on Grey Wolf Optimization and Recurrent Neural Network" was retracted in 2023. Reasons: suspected computer-generated content; unreliable results or conclusions; concerns about the data; concerns about the results or conclusions.

### 4.1. In-Demand Analytics Skills

In demand analytics skills, we assessed the employee experience, people analysis, internal recruiting, and multigenerational workforce. The in-demand analytics skills are depicted in Figure 4.

Figure 4 explains employee experience with a score of 94 percent, people analytics with a score of 85 percent, internal recruitment with a score of 82 percent, and a multigenerational workforce with a score of 74 percent. While comparing the employee experience, people analytics, and internal recruiting with a multigenerational workforce, it is shown that the multigenerational workforce is lower than the others.

### 4.2. Human Resource Satisfaction Index (HRSI)

In HRSI, we assessed the employer image, employee expectations, perceived HR service quality, value perceived by the employee, employee satisfaction, employee loyalty, and HRSI. The human resource satisfaction index is depicted in Figure 5.

Figure 5 shows employer image with a score of 34.94 percent, employer expectations with a score of 51.62 percent, perceived HR service quality with a score of 71.35 percent, value perceived by the employee with a score of 70.43 percent, employee satisfaction with a score of 54.45 percent, employee loyalty with a score of 42.23 percent, and HRSI with a score of 54.17 percent. While comparing employer image, employer expectations, perceived HR service quality, employee satisfaction, employee loyalty, and HRSI, it is shown that perceived HR service is higher than the others.

### 4.3. Prediction Rate

In other words, if an early warning system can accurately predict a need for HR, then it has a high predictive value.  Figure 6 represents the prediction rate.

In Figure 6, we evaluate the convolutional neural network with a prediction rate of 73 percent, the double cycle neural network with a prediction rate of 63 percent, the whale optimization with a prediction rate of 85 percent, and the particle swarm optimization with a prediction rate of 58 percent, and we propose RNN + GWO with a prediction rate of 95 percent. The results of the comparisons reveal that the suggested approach is superior to each of the four methods that already exist.

### 4.4. Error Rate

It is the percentage of incorrect units of data transferred in comparison to the overall number of units of data.  Figure 7 shows the error rate.

In Figure 7, we evaluate the convolution neural network with an error rate of 93 percent, the double cycle neural network with an error rate of 85 percent, the whale optimization with an error rate of 80 percent, and the particle swarm optimization with an error rate of 75 percent, and we propose RNN + GWO with an error rate of 50 percent. The results of the comparisons demonstrate that the suggested approach is inferior to each of the four other strategies already in use.

The article "Human Resource Demand Prediction and Configuration Model Based on Grey Wolf Optimization and Recurrent Neural Network" was retracted in 2023. Reasons: suspected computer-generated content; unreliable results or conclusions; concerns about the data; concerns about the results or conclusions.

## 5. Discussion

In CNN (existing), this model presents several problems, the most significant of which are overfitting, inflating gradients, and class unbalances. The effectiveness of the model may suffer as a result of these concerns. Negative aspects of the DCNN (existing) include the following: the lifetime of the network is uncertain; the working of the network is not described, and it is difficult to demonstrate the issue to the network. The whale optimization (existing) suffers from some flaws, the most notable of which are its sluggish convergence, poor solution accuracy, and the ease with which it might fall into the local optimum solution. The particle swarm optimization (PSO) technique has several drawbacks, the most notable of which are that it is simple to become stuck in a local optimum in a high-dimensional space and that it has a slow convergence rate throughout the repeated process.

## 6. Conclusion

The key to an enterprise's long-term success is its ability to effectively use its HR. There will be a great amount of data on HR created inside the firm as the company continues to grow and expand. Data on corporate HR are often inadequate or inaccurate since the demand for HR is impacted by so many factors. As a result, there is a high degree of nonlinearity between various components and demand for HR. Human resource demand may be forecasted using a recurrent neural network (RNN) and grey wolf optimization (GWO) which is a revolutionary quantitative forecasting approach of tremendous theoretical significance. The first step is to get the data and normalize it. Principal component analysis (PCA) is used to identify the characteristics, and the suggested RNN with GWO can accurately estimate human resource requirements. To make forecasting more relevant, flexible, and accurate, the human resource demand prediction model was developed and it might help organizations better manage their HR to meet their priorities. El Health employs IoT sensors in particular to monitor employee demand, which is analyzed as a time-series data and utilized to forecast future need.

## Figures and Tables

**Figure 1:** Human resource planning.

**Figure 2:** Overall methodology used.

**Figure 3:** Framework of RNN.

**Figure 4:** In-demand analytics skills.

**Figure 5:** Human resource satisfaction index (HRSI).

The article "Human Resource Demand Prediction and Configuration Model Based on Grey Wolf Optimization and Recurrent Neural Network" was retracted in 2023. Reasons: suspected computer-generated content; unreliable results or conclusions; concerns about the data; concerns about the results or conclusions.

**Figure 6:** Comparative analysis of prediction rate for suggested and traditional methods.

**Figure 7:** Comparative analysis of error rate for suggested and traditional methods.

**Algorithm 1:** Grey wolf optimization (GWO).

## Data Availability

No data were used in this study.
